The article "A Study of Fiscal Expenditure Structure and Green Economic Growth Effects: A Sample from Asian Economies" was published in 2022. Journal: J Environ Public Health.

# A Study of Fiscal Expenditure Structure and Green Economic Growth Effects: A Sample from Asian Economies

**DOI:** 10.1155/2022/2180532

**Published:** 2022-09-22

**Authors:** Chi Gong, Yizi Wan

**Affiliations:** School of Economics, Sichuan University, Chengdu, Sichuan 610041, China

## Abstract

The structure of fiscal expenditure in China has been suffering from over-reliance on a single type, while synchronisation and coordination with economic growth are lacking. This paper studies and analyses fiscal expenditure and green from a theoretical perspective. There is a close link between the structure of fiscal expenditure and green economic growth, and a reasonable and appropriate selection and allocation is conducive to promoting the overall development level of China, while financial resources input is a key consideration in optimising the structure of fiscal expenditure. This paper proposes hypotheses and establishes a regression model after an in-depth study of fiscal expenditure in a provincial economy in Asia in the light of domestic and international literature. Through empirical analysis, a green GDP reflecting economic growth and environmental pollution is synthesised using the principle of output per unit of pollution, and the impact of fiscal expenditure structure on green economic growth in China is empirically tested.

## 1. Introduction

The structure of fiscal expenditure has been a hot issue for scholars both at home and abroad and has been analysed and discussed in great depth. However, the government as a public good has the characteristics of non-competitiveness and exclusivity: firstly, it has the same indivisibility as other commodities; secondly, it is a form of public service supply or service supply; finally, there are two main sources of finance for fiscal expenditure: one is the central and local budget allocation, and the other is provided through tax revenue [1]. However, in the process of reform and opening up, many new problems have emerged. For example, the lack of investment in the “three rural areas,” the backwardness of rural infrastructure construction and a series of other problems have plagued the process of economic development, and the problem of financial resources has become increasingly prominent. At the same time, as the level of social productivity increases [2], China's consumption of natural resources continues to intensify and other factors lead to serious environmental pollution and waste of resources, which seriously restrict our green economy and sustainable development. The consequences of the unreasonable structure of fiscal expenditure, such as the waste of resources and low utilisation rate, are already unimaginable. Therefore, how to adjust and optimise the relationship between fiscal expenditure structure and green GDP has become one of the hot spots of current research [3].

The article "A Study of Fiscal Expenditure Structure and Green Economic Growth Effects: A Sample from Asian Economies" was published in 2022. Journal: J Environ Public Health.

Fiscal expenditure has always been the top priority of China's economic development, playing an important role in promoting social equity and resource allocation, as well as being of great significance to the achievement of scientific and sustainable development in China. However, in recent years [4], the government has been increasing its efforts in environmental protection to strengthen environmental protection and ecological construction. The 12th Five-Year Plan for Energy Conservation and Emission Reduction was officially implemented on 1 May 2016, and the introduction of green fiscal policies was adopted [5].

The structure of fiscal expenditure refers to the allocation of funds by the national government within a certain period of time, which reflects the allocation of various resources and the proportional relationship between various economic factors in the process of social reproduction. With the rapid development of China's economy, fiscal expenditure is becoming more and more important in the national economy, but at the same time, there are also many problems [6]. As environmental pollution, resource waste and ecological damage are becoming increasingly serious, and how to achieve sustainable solutions to these problems has become a new issue facing the government. This paper argues that there is a link between green economic growth and the structure of fiscal expenditure as follows: the two have different degrees of impact on income and employment. The former measures the overall development of a region or industry in terms of total GDP, while the latter reflects a country's position and role in the national economy through the direct and indirect effects of national fiscal revenues as a percentage of gross national product (GNP) [7]. This paper analyses the relationship between green fiscal policy and industrial structure to understand the current trends in industrial structure and to discover what factors have influenced the current state of China's economic development and the future direction of economic development, and on this basis to propose corresponding optimisation measures to better promote the coordination of China's overall social, environmental, resource, and ecological benefits [8–10].

## 2. Analysis of the Factors Influencing the Promotion of Green Economic Growth

### 2.1. Analysis of the Mechanism for Promoting Green Economic Growth

In the past economic growth process, people generally focus more on the cycle between the economic system and the social system, but less consider the virtuous cycle between the economy, society, and the ecosystem. This phenomenon is evident in both theory and practice, for example, the Douglas production function, the endogenous economic growth model, the Solow economic growth model, and other classical growth models do not consider the contribution of ecosystems to economic growth. In practice, under the market mechanism, it is difficult for the economic system to spontaneously form a reasonable compensation mechanism for the ecosystem. Under the crude economic growth model, the dependence of economic growth on the inputs of ecological factors is higher, and the degree of damage to ecosystems is more serious. The negative feedback force between the economic and social systems and ecosystems is more obvious, and this imbalance leads to development that is not sustainable. As shown in Figure 1, it is generally accepted that the social system contributes to the growth of the economic system by providing labour and investment, and the economic system raises people's material living standards by providing goods and services.

The article "A Study of Fiscal Expenditure Structure and Green Economic Growth Effects: A Sample from Asian Economies" was published in 2022. Journal: J Environ Public Health.

The above diagram shows that economic growth is the result of joint inputs from social and ecological systems. The ecosystem provides ecological factors and services, and the social system provides labour and capital, which together contribute to economic growth. In turn, economic growth provides goods and services to the social system without providing positive feedback to the ecosystem, making it difficult for the ecosystem to be reasonably compensated. At the same time, there are also negative feedbacks between the social system and the ecosystem [11]. The pollutants and wastes produced by society in the process of consuming goods and services will cause further degradation of the ecosystem and impede social development. This deterioration of the ecosystem will also result in a reduction in the “quality” and “quantity” of ecological factors and services available from the ecosystem, which will impede economic growth and lead to a reduction in the goods and services available from the economic system, thus creating a vicious circle [12].

There are both negative and positive feedback mechanisms between the three systems. Only by forming a positive feedback mechanism between the three systems can a balanced development be achieved and the three systems can co-exist and jointly promote green economic growth. First, the positive feedback relationship between the economy and the ecosystem. Ecological factors and services are input into the economic system and are the basis for economic growth. At the same time, economic growth creates a material base, a level of science and technology that can repair and rebuild ecosystems and can enhance the ability of ecosystems to cycle through to provide ecological factors and services. Secondly, there is a positive feedback relationship between social systems and ecosystems. The social system has human development as its main goal, and the improvement of the comprehensive quality of human beings is conducive to people raising their awareness of environmental protection, improving their level of science and technology, and contributing to the protection and repair of the ecological environment [13]. On the other hand, the ecological environment is also the basis for people's survival and life, so the good or bad ecological environment is the basis for social development. Thirdly, there is a positive feedback mechanism between the economic and social systems. On the one hand, the economic system is the basis of human development and is the foundation of social development. The development of the economic system is the basis for social development. Economic growth is both the basis for human material life and makes it possible to improve education and scientific and technological innovation, thus promoting social progress. On the other hand, social development can also contribute to economic development. Social conditions such as social harmony, fair distribution, effective forms of cooperation, and highly qualified human resources are more conducive to driving economic growth [14]. As shown in Figure 2, the three systems can either constrain or reinforce each other and develop together.

The article "A Study of Fiscal Expenditure Structure and Green Economic Growth Effects: A Sample from Asian Economies" was published in 2022. Journal: J Environ Public Health.

Thus, there is a mutual feedback mechanism between the three systems. The ecosystem is the basis for development, while there are also positive and negative feedback effects of economic system development on the social and ecological systems. Green economic growth is not the absence of economic development, but the formation of positive economic, social, and ecological feedback mechanisms.

### 2.2. Using the Cobb-Douglas Production Function to Construct a Green Economic Growth Model

The classical Cobb-Douglas production function considers only the amount of capital and labour inputs, and the Cobb-Douglas production function is as follows.

(1) $$\begin{array}{c} Y=AL^{\alpha }K^{\beta }. \end{array}$$

*Y* represents the quantity of output, *A* represents the total factor productivity, *L* represents the quantity of labour, *K* represents the quantity of capital, and *α* and *β* represent the elasticity of labour and capital to output, respectively, 0 < *α* and *β* < 1.

Green economic growth is people-centred development, a balanced development of ecosystems, social systems, and economic systems. The Douglas production function, which includes ecological occupation, means that the level of labour, capital, and ecological factor inputs determines the level of output of the economy at a certain total factor productivity. Ecological factors, as one of the driving forces of economic growth, should be included in the Douglas production function. The Douglas production function with ecological occupation is as follows: assume that the annual ecological factor input is *E*1 and *γ* indicates the elasticity of ecological occupation with respect to output, 0 < *γ* < 1.

(2) $$\begin{array}{c} Y=E_{1}^{\gamma }AL^{\alpha }K^{\beta }. \end{array}$$

The progressive aspect of *E*1, together with *L* and *K*, as an input factor for economic growth is that the ecological factor input is not an output of labour and capital, but a primitive input factor parallel to labour and capital, which represents when the ecological factor is not fully regenerative, not constantly regenerative by the increase in the amount of labour and capital. The economy is not constantly increasing in production only by increasing the amount of labour and capital.

The article "A Study of Fiscal Expenditure Structure and Green Economic Growth Effects: A Sample from Asian Economies" was published in 2022. Journal: J Environ Public Health.

### 2.3. Accounting for the Costs of Economic Growth and Growth Models that Incorporate Green Economic Growth Mechanisms

It is generally accepted that economic growth and social consumption lead to an increase in ecological occupation and thus in the cost of development. On the one hand, an increase in the ecological inputs required in the process of economic growth leads to an increase in ecological occupation. On the other hand, the increase in pollutants and waste generated by economic production and social consumption leads to an increase in ecological occupation. The increase in ecological occupation not only increases ecological costs but also social costs. Ecological occupation and the ecological environment are negatively related. When ecological occupation exceeds ecological carrying capacity, the ecological environment will be damaged, i.e., an increase in ecological occupation will lead to a decrease in the total ecological environment, a decrease in the ecological elements and ecological services available in the ecological environment, and an increase in ecological costs. The destruction of the ecological environment will lead to a series of social problems, such as an increase in the incidence of cancer and lung disease, which will lead to a further increase in social costs. Assuming that the total ecological environment is *TE*, the relationship between ecological occupation and ecological environment is as follows.

(3) $$\begin{array}{c} {TE}_{1}={TE}_{0}-ef\left(E\right)+∆E\left(i\right). \end{array}$$

*TE*0 represents the total ecological environment in the previous period, *TE*1 represents the total ecological environment in the current period, and *ef*(*E*) represents the degree of influence of the level of ecological occupation on the total ecological environment. *ef* functions are influenced by factors such as production patterns, consumption patterns, the degree of ecological dissipation of pollutants and waste, the ability of science and technology to degrade pollutants, and the carrying capacity of ecosystems. *e* represents the level of ecological occupation and is equal to the ecological factor input (*E*1) and the sum of the inputs of pollutants and waste dissipation (*E*2). Δ*E*(*i*) represents the impact of ecological restoration inputs on the total ecological environment, which is influenced by the level of science and technology to combat pollution and the expenditure on protecting and restoring ecosystems (*i*). Therefore, when the amount of ecological restoration is 0, and the ecological occupation is greater than the ecological carrying capacity, i.e., greater than what the ecosystem can consume through its own cycle, *ef*(*E*) is greater than 0, the total ecological environment is reduced, and *TE*1 is less than *TE*0.

The article "A Study of Fiscal Expenditure Structure and Green Economic Growth Effects: A Sample from Asian Economies" was published in 2022. Journal: J Environ Public Health.

Studies have shown that a reduction in the total ecological environment will result in a reduction in the ecological services available, further increasing the cost to society. When the total ecological environment is reduced, the ecological services available to people are also reduced. For example, fossil energy burning leads to high levels of haze, further leading to people not being able to breathe fresh air and creating or increasing the cost of access to health care. In some places, land cannot be cultivated due to mining and water sources are contaminated and undrinkable, increasing social costs such as access to health care and migration. The reduction in the total ecological stock thus brings increased costs to society in two ways. Firstly, the deterioration of the ecological environment increases the social costs of medical care, ecological services, and migration for people. The higher the economic level of a country or a region, the greater the impact of a smaller ecological stock on the level of social well-being. Secondly, people's input costs to restore the ecological environment, including economic costs and human costs.

(4) $$\begin{array}{c} C=cf\left({TE}_{1}\right)+i+C_{0}. \end{array}$$

*C* represents the total cost, assuming that the ecosystem is an ecological asset that can be converted into a corresponding output for comparison. The *cf* function represents the effect of the total ecosystem on the total cost. If the total ecological environment is low, or if the ecological carrying capacity is low, or if the ecological input and consumption capacity is lower, this will lead to limited economic growth, resulting in higher economic costs. On the other hand, a lower total ecological environment means that the ecological elements and ecological services that the ecological environment can provide will also be lower, resulting in higher social costs. Therefore, a reduction in the total ecological environment will lead to an increase in economic and social costs. *i* represents the expenditure in a country's economy that is invested in ecological protection and restoration.

The article "A Study of Fiscal Expenditure Structure and Green Economic Growth Effects: A Sample from Asian Economies" was published in 2022. Journal: J Environ Public Health.

Bringing equation (3) and equation (4) into equation (2) yields a Douglas production function that includes social and ecological costs as follows.

(5) $$\begin{array}{c} R=AL^{\alpha }K^{\beta }E_{1}^{\gamma }-cf\left[TE_{0}-ef\left(E\right)+∆E\left(i\right)\right]-i-C_{0}. \end{array}$$

The analysis from the formula has the following implications:

Firstly, analysed in terms of the impact of the economic system in the development process, i.e., from A1, promoting green production has the following implications, firstly increasing the level of science and technology innovation, i.e., increasing the total factor productivity of production and obtaining maximum economic output with limited ecological factor inputs; secondly, green economic growth can increase the contribution of labour (*L*) and capital (*K*) to the economic system and reduce the dependence on the ecosystem. Second, green economic growth can increase the contribution of labour (*L*) and capital (*K*) to the economic system and reduce dependence on the ecosystem. Thirdly, it reduces ecological factor inputs (*E*1), especially those that are not recycled.

Secondly, the social cost of ecosystem damage during development is analysed in terms of the *cf* [*TE*0 − *ef*(*E*) + Δ*E*(*i*)] function, i.e., the better the ecosystem, the lower the social cost, with an inverse relationship between the two. The total ecological environment is influenced by the original ecological stock, ecological occupancy flow, and ecological restoration. The higher the value of ecological restoration construction, the less ecological occupation, the higher the total ecological environment (TE1), and the higher the ecological carrying capacity. Secondly, the level and scope of ecological restoration construction by ecological conservation inputs (*i*) can be improved through scientific and technological development, and the maximum amount of ecological restoration can be obtained with limited ecological conservation inputs. Thirdly, from the analysis of the ecosystem, promoting the development of the ecosystem requires an increase in expenditure on ecological inputs (*i*).

The article "A Study of Fiscal Expenditure Structure and Green Economic Growth Effects: A Sample from Asian Economies" was published in 2022. Journal: J Environ Public Health.

Finally, from the analysis of the economic system, the social system and the synergistic development of the ecosystem, when the economic level is high and the total amount of ecological environment is low, the higher the cost of the total amount of ecological environment to the social system in the cf function; when the building capacity of ecological restoration is high, the more the increase of the economic system's input to the total amount of ecosystem. In terms of the contribution of ecosystems to economic systems, increasing ecological carrying capacity can increase the contribution of ecologically occupied economic systems. Therefore, the promotion of green economic growth should increase the efficiency of the output of ecological occupation, the capacity of ecological restoration, and the increase of ecological carrying capacity.

## 3. A Test of the Impact of Fiscal Expenditure Structure on Green Economic Growth

Compared to Western federalism, the Chinese style of fiscal expenditure structure reform focuses more on incentivising local governments to focus on economic growth. Although the fiscal expenditure structure has brought about the phenomenon of “beggar-thy-neighbour” and rent-seeking corruption, it has generally contributed to the growth of the regional economy and is an important factor in driving China's high economic growth. In addition to financial incentives, the promotion mechanism for officials has motivated local governments to promote economic growth. China has a top-down vertical management system and a strict system of mobility control, so the Western “voting with one's feet” does not work substantially in China. In China's multilayered commissioning relationship, economic performance assessment is the main indicator for evaluating the performance of officials in office, and some studies have shown a positive correlation between the promotion opportunities of officials and regional economic performance. In summary, there are two types of competition between local governments: one is for regional economic growth and fiscal revenue, and the other is for political promotion. Either type of competition must be obtained through economic growth performance; therefore, the fiscal expenditure structure and competition between governments drive economic growth. The Chinese-style fiscal expenditure structure drives economic growth while also having an impact on the environment. The green economic growth studied in this paper is a kind of economic growth that only considers the environmental pollution status. Therefore, when the fiscal expenditure structure policy affects the economic growth and also has an impact on the environmental pollution status, it will inevitably bring some impact on the green economic growth, and the specific impact depends on the direction and size of the impact of the fiscal expenditure structure on the environmental quality when driving the economic growth. If the structure of fiscal expenditure exacerbates environmental pollution while driving economic growth, and the economic growth brought about is not enough to compensate for the cost of environmental pollution, then the structure of fiscal expenditure will have a suppressive effect on green economic growth; if the structure of fiscal expenditure exacerbates environmental pollution while driving economic growth, but the increase in economic growth can compensate for the cost of environmental pollution, then the structure of fiscal expenditure has a suppressive effect on green If the fiscal expenditure structure contributes to the improvement of environmental pollution while driving economic growth, then the implementation of the fiscal expenditure structure contributes to green economic growth, and this green growth effect is greater than the economic growth effect. Based on the above analysis, this paper constructs a comprehensive index to reflect the environmental pollution situation, and empirically analyses the impact of the fiscal expenditure structure on environmental pollution, and tests whether the fiscal expenditure structure has an ameliorating effect on environmental pollution or a counter-effect of aggravating it. The paper then uses the comprehensive index of environmental pollution and GDP to synthesise green GDP, which reflects the cost of environmental pollution, and uses green GDP to measure green economic growth.

The article "A Study of Fiscal Expenditure Structure and Green Economic Growth Effects: A Sample from Asian Economies" was published in 2022. Journal: J Environ Public Health.

### 3.1. Measurement of Green Economic Growth

Green economic growth is a sustainable form of economic growth, which can reconcile economic development with resources and environment and, to a certain extent, achieve the organic unity of economic development, environmental protection, and ecological environment improvement.

This paper uses the term “green GDP” (i.e., EDP) to refer to the economic growth rate. In this paper, we use green GDP (i.e., EDP) to measure China's green economic growth. Based on the summary of previous studies, we draw on the measurement method of [15] and use the comprehensive index of environmental pollution constructed in Chapter 3 to construct the green output index of EDP by adopting the principle of output per unit of pollution, whose mathematical expression is EDP = GDP/comprehensive index of environmental pollution. The lower the EDP index and the larger the GDP, the higher the quality of economic growth and the higher the level of green economic development. This paper uses the real EDP per capita growth rate calculated by the growth rate definition formula to measure green economic growth, which does not reflect the full range of green economic development, but it is considered a useful attempt to portray the level of green economic development using EDP per capita until a better comprehensive indicator is available. Green economic growth is expressed as the growth rate of EDP, with the following formula.

(6) $$\begin{array}{c} \text{EDP}=\frac{\text{ED}{\text{P}}_{it}-\text{ED}{\text{P}}_{i,t-1}}{\text{ED}{\text{P}}_{i,t-1}}. \end{array}$$

### 3.2. Variable Setting and Descriptive Statistical Analysis

This paper studies the impact of fiscal expenditure structure on green economic growth and therefore sets green economic growth (edp) as the explanatory variable. In order to compare the similarities and differences between the impact of fiscal expenditure structure on green economic growth (edp) reflecting environmental costs and economic growth (gdp) without considering environmental costs, economic growth (gdp) is chosen as the explanatory variable in this paper. The data used in this study were obtained from the Wind database and the WIEGO statistical database. The sample data was selected from 30 provinces in China over a 14-year period, and the total cumulative sample size was 408, excluding vacant values. The results of the descriptive statistical analysis of the selected data are shown in Table 1.

### 3.3. Analysis of Regression Results Based on a Random Effects Model

In order to study the impact of fiscal expenditure structure on green economic growth, this paper conducts an econometric analysis of panel data and the basic regression model is set as

(7) $$\begin{array}{c} \text{ed}{\text{p}}_{ii}=\alpha_{1}+\beta_{1}\text{De}{\text{c}}_{ii}+\beta_{2}\text{FD}{\text{I}}_{ii}\times \text{Ex}{\text{p}}_{ii}+\beta_{3}k_{ii}+\beta_{4}En_{ii}+\beta_{5}Is_{ii}+\beta_{6}\text{Jrbe}{\text{n}}_{ii}+\varepsilon_{ii}. \end{array}$$

The *F*-test and Hausman test were used to select between the mixed model, the fixed-effects model, and the random effects model to find the most suitable regression model for the regression analysis.

#### 3.3.1. *F*-Test

The *F*-test is used to determine whether the assumption of parameter constraint is valid by comparing the squared residuals of the regression of the fixed-effects model with constraints to the squared residuals of the regression of the fixed-effects model without constraints. The results of the *F*-test are shown in Table 2.

The article "A Study of Fiscal Expenditure Structure and Green Economic Growth Effects: A Sample from Asian Economies" was published in 2022. Journal: J Environ Public Health.

The test results showed that with *P* ≤ 0.001, regardless of expenditure as the explanatory variable, and thus rejecting the null hypothesis at a 1% significance level, the fixed-effect model outperformed the mixed regression model.

#### 3.3.2. Hausman Test

In order to compare which of the random effects model and the fixed-effects model is more applicable to this panel data, the Hausman test was further conducted and the results of the test are shown in Table 3.

The Hausman test results show that the random effects model hypothesis cannot be rejected at the 1% significance level, so the random effects model is used to regress the panel data. In this paper, a random effects model regression was conducted on the panel data using stata12.0 to investigate the impact of fiscal expenditure structure on green economic growth. The regression results are shown in Table 4.

The regression results show that there is a significant positive relationship between fiscal expenditure and green economic growth. For the study on the influence of control variables on green economic growth, the influence of per capita fixed capital growth rate on green economic growth is significantly positive, indicating that among the factors promoting green economic growth, fixed capital investment plays a great role; the influence of industrial structure is significantly positive; a reasonable explanation for this phenomenon is that the green economic growth in this paper is the growth rate of output per unit of pollution, although the secondary industry is the most polluting industry. Although the secondary sector is the most polluting industry, it is also the main driver of economic growth, and the contribution of the secondary sector to economic growth can compensate for the cost of environmental pollution, so the effect of industrial structure is positive overall. The above findings do not obscure the fact that the secondary sector also contributes to environmental pollution, so the government needs to guide such industries to use advanced production technologies to reduce pollutant output and to strengthen the regulation of pollutant compliance to facilitate the transformation of the secondary sector's production methods. The significant negative effect of resource endowment is due to the fact that, for the time being, labour-intensive industries are more advantageous than capital-intensive industries, and capital-intensive provinces tend to be accompanied by lower technical efficiency.

### 3.4. Comparative Analysis of Differences in the Economic Effects of Fiscal Expenditure with and without Environmental Constraints

In order to compare the similarities and differences in the effects of fiscal expenditure structure on green economic growth (edp), which reflects environmental costs, and economic growth (gdp), which does not take into account environmental costs, the regression results are shown in Table 5.

The article "A Study of Fiscal Expenditure Structure and Green Economic Growth Effects: A Sample from Asian Economies" was published in 2022. Journal: J Environ Public Health.

In order to compare the similarities and differences in the effects of fiscal expenditure structure on green economic growth (edp) reflecting environmental costs and economic growth (gdp) without considering environmental costs, regressions were also conducted on fiscal expenditure structure and economic growth.

#### 3.4.1. Direct Impact of Fiscal Expenditure Structure

From the regression results, it can be seen that the structure of fiscal expenditure has a significant positive relationship with green economic growth and economic growth. From the magnitude of the regression coefficients, the coefficient of the impact of fiscal expenditure structure on green economic growth is larger than that on economic growth, which echoes the findings of the study on the impact of environmental pollution: the direct impact of fiscal expenditure structure on environmental pollution is negatively related, i.e., the improvement of fiscal expenditure structure helps to improve environmental pollution. While boosting economic growth, it also improves environmental pollution, so the impact of fiscal expenditure structure on green economic growth is greater than the impact on economic growth.

#### 3.4.2. Indirect Effects of Fiscal Expenditure Structure

The coefficient of the cross-section of fiscal expenditure structure and FDI variables on economic growth is significantly positive, while the coefficient of the cross-section of revenue decentralisation and FDI variables on economic growth is negative but insignificant. The explanation for this phenomenon draws on the findings of [16], where there is a threshold effect based on the degree of fiscal expenditure structure in the case of technology spillovers from FDI. When the level of fiscal expenditure is too low, local governments are competing for FDI by attracting foreign capital through tax incentives on the one hand, and on the other hand, based on the pressure of fiscal expenditure, part of the basic inputs are not guaranteed, hindering domestic enterprises. When the level of fiscal expenditure is relatively high, local governments are able to improve the local investment environment and increase their incentive to fully absorb the spillover effects of FDI and improve local productivity. The level of fiscal expenditure in China is much higher than the level of fiscal revenue, thus leading to the phenomenon that the coefficient of the cross-section of fiscal expenditure structure and FDI variables on economic growth is significantly positive, while the coefficient of the cross-section of revenue decentralisation and FDI variables on economic growth is negative but not significant.

The article "A Study of Fiscal Expenditure Structure and Green Economic Growth Effects: A Sample from Asian Economies" was published in 2022. Journal: J Environ Public Health.

The cross-section of fiscal expenditure structure and FDI variables has a negative but insignificant coefficient on green economic growth, while the cross-section of revenue decentralisation and FDI variables has a significantly negative coefficient on green economic growth. The explanation for this phenomenon is that, combined with the findings of this paper on the relationship between fiscal expenditure structure and environmental pollution, the fiscal expenditure structure intensifies competition among governments, and government competition for FDI brings about distorted government behaviour, which brings about environmental pollution; under the fiscal expenditure structure measured by the fiscal expenditure structure, the fiscal expenditure structure encourages local enterprises to absorb FDI technology spillovers, which increases productivity However, this increase in productivity is not sufficient to compensate for the cost of environmental pollution, and therefore, with the introduction of FDI, the contribution of the fiscal expenditure structure to green economic growth is weakened; under the fiscal expenditure structure measured by income decentralisation, the fiscal expenditure structure hinders the absorption of FDI technology spillovers by local enterprises, which does not increase productivity and brings about pollution at the same time, which makes the impact of the cross multiplier on green growth significantly negative " the fiscal expenditure structure... fiscal expenditure to green growth." with:the structure of fiscal spending discourages local firms from absorbing foreign investment and technology, affects productivity, and is detrimental to environmental protection, while making the cross multipliers significantly negative for green growth, i.e., the low level of fiscal spending structure weakens the contribution of fiscal spending to green growth.

In general, a good expenditure structure can facilitate the absorption of FDI technology spillovers by local enterprises and increase economic growth. As long as the “competition among governments” is addressed, the environmental threshold is not lowered and environmental regulation and management are strengthened, the quality of economic growth can be improved and green economic growth can be driven.

## 4. Policy Recommendations

In the empirical analysis of fiscal expenditure structure and green economic growth, we can find that although China has become the world's largest consumer market, there are still many improvements to be made and more options to choose from that affect its efficiency in resource allocation and environmental quality. Therefore, we propose policy recommendations at three levels: inter-governmental, intra-enterprise, and external.

The article "A Study of Fiscal Expenditure Structure and Green Economic Growth Effects: A Sample from Asian Economies" was published in 2022. Journal: J Environ Public Health.

### 4.1. Implement Structural Fiscal Expenditure Policies

First, clarify the division of fiscal and administrative powers between the central and local governments and improve the economic efficiency of government transfers. Financial power refers to the power of governments at all levels to obtain fiscal revenues and allocate fiscal expenditures, as well as the right to own and manage local wealth. Affairs power, on the other hand, refers to the function of governments at all levels to carry out their basic duties, to manage regional administration and economy, and to provide public goods and public services. The two are both distinct from each other and complementary to each other. Financial power is the material basis for the realisation of the government's powers, which in turn provides the criteria and basis for the exercise of financial power. Under the current system of fiscal decentralisation in China, the division of responsibilities between central and local financial and ministerial powers is unclear, local governments rely excessively on central transfer payments for their sources of income, and there is a huge gap between local financial revenues and expenditures. In the long run, this is not conducive to the healthy development of our economy and society. Therefore, we should start by promoting the reform of the structure of fiscal affairs and financial powers to improve the efficiency of fiscal expenditure.

Secondly, we should increase investment in science and technology innovation, support the development of strategic emerging industries and service industries, and provide sustained impetus for the healthy development of our economy. Striving to improve the capacity of independent innovation, relying on innovation and entrepreneurship to expand the scale of employment and raise people's income, and promoting the transformation and upgrading of China's industrial and economic structures are important tasks for China's economic development at present. While the main actors in improving the capacity for independent innovation and developing new industries are the market, enterprises, and the people, government intervention and adjustment is also one of the essential conditions for their healthy development. Among the many ways of government regulation and control, fiscal expenditure policy is of particular significance. On the one hand, the government, with its strong economic power, can provide the necessary upfront capital for the development of the relevant industries and improve market confidence. On the other hand, government spending has a strong guiding and demonstration effect. Increasing government investment in science and technology innovation can lead to a greater convergence of idle social capital in new industries and increase the enthusiasm of the whole society for innovation and entrepreneurship. Therefore, we should shift the fiscal expenditure towards the field of science and technology innovation, play the guiding role of fiscal expenditure, increase the investment in research and development in key areas and core technologies, focus on cultivating a number of products and enterprises that can independently master the core technologies, have high added value of products and have international competitiveness, and play its demonstration effect. At the same time, more special funds should be set up for R&D in science and technology innovation, more investment should be made in the construction of relevant science and technology industrial parks, and more financial subsidies should be provided for the production and operation of strategic emerging enterprises. Of course, we should also be aware that the excessive use of government financial subsidies also has the disadvantage of distorting market prices. For this reason, we can appropriately introduce a competition mechanism into our fiscal subsidy policy, make timely and dynamic adjustments to the scope and intensity of fiscal subsidies according to the actual situation of industrial development, optimise the structure of fiscal expenditure subsidies, improve the economic efficiency of fiscal expenditure, and provide a favourable policy environment for the development of relevant industries.

The article "A Study of Fiscal Expenditure Structure and Green Economic Growth Effects: A Sample from Asian Economies" was published in 2022. Journal: J Environ Public Health.

Thirdly, we should strengthen investment in people's livelihood, ease social conflicts, and create a favourable social environment for the smooth operation of the economy. Premier Li Keqiang has pointed out that continuous improvement of people's livelihood is one of the objectives of our government's administration. He believes that the government should strive to become a government of people's livelihood, focusing on safeguarding basic livelihoods and gradually filling up the shortcomings of people's livelihoods such as compulsory education, healthcare, and retirement.

### 4.2. Reducing the Scale of Government Maintenance Expenditure

First, the reform of administrative institutions should be further deepened, government agencies should be streamlined, and government administrative expenditure should be vigorously reduced. First, we should strengthen the innovation of government organisations and deepen the reform of administrative institutions. We should implement the 2018 State Council's institutional reform programme, which, on the one hand, should reflect the reform idea of one department being responsible for one thing, integrate departments and institutions with similar functions, continuously optimise the setting of administrative institutions, and reduce institutional overlap. On the other hand, government functions should be redefined and new departments formed in accordance with the real needs of national and social development in the new era. We should scientifically dismantle and integrate government administrative agencies and strive to build a modern government organisation system with unified powers and responsibilities, a clear division of labour, efficient operation, public rationality, and adaptability to the needs of the new era. Secondly, we should change the original rough and tumble system. Secondly, we should change the original rough and loose way of controlling government administrative expenses, set clear objectives and standards for controlling administrative expenses, increase the control of each unit's budget, further clarify and implement the responsibility system for expenses, and realise strict management and effective monitoring of government administrative expenses. At the same time, it should also further enhance the cost consciousness and saving awareness of all administrative and institutional units, in line with the principle of living within one's means and practising economy, to continuously reduce administrative costs and build an economical government.

Second, further simplify and decentralise government and continue to reduce government approvals. Simplify and decentralise government and reduce government intervention in market activities.

In addition to enhancing market dynamics, it will also significantly reduce the scale of government administrative expenditure in related areas.

This will be beneficial to the role of the market mechanism and promote the smooth operation of the economy. Therefore, we should further.

We should further accelerate the pace of decentralisation and simplification of government administration, except in strategic areas such as energy and minerals, which are of national importance and livelihood. Simplify the administrative approval procedures for normal production and operation and enhance the vitality and autonomy of the market. At the same time, the government should. At the same time, we should thoroughly implement the directives of the 18th Party Congress and establish and improve the negative list and power list system for government investment projects, and the powers and responsibilities of the government should be further clarified, and the powers and scope of the government's administrative approvals should be clearly disclosed to society as a whole and subject to the supervision and questioning of society as a whole.

The article "A Study of Fiscal Expenditure Structure and Green Economic Growth Effects: A Sample from Asian Economies" was published in 2022. Journal: J Environ Public Health.

Thirdly, we should speed up the innovation of government administration, reduce government administrative costs, and improve the efficiency and level of government macro-control. Innovation in government administration can effectively reduce administrative costs and streamline administrative expenses, while at the same time effectively improving the efficiency of governance and realising scientific and effective governance of society by the government. Therefore, we should vigorously innovate government administration and promote the process of modernising the government's ability to govern.

### 4.3. Maintain the Stability of Social Service Expenditure Policies

A stable and continuous fiscal expenditure policy can provide a good policy environment for the development of economic agents, which is conducive to the formation of rational market expectations by market agents and the reduction of market speculation brought about by unstable policies, which is beneficial to the stability and healthy development of the macro economy. Therefore, we should attach importance to maintaining the stability of fiscal expenditure, especially social service expenditure policies, to enhance the efficiency of government macro-control. People's livelihood-oriented fiscal expenditure policies should be stable, and innovation-oriented fiscal expenditure policies should be continuous. Only by ensuring the continuity of these policies in time and space can we guide the market investment and production subjects to establish rational policy expectations, increase the enthusiasm of market subjects for “dual innovation,” and encourage relevant enterprises and investors to make long-term strategic decisions, so as to reduce the negative impact of market speculation on the stable and healthy development of the economy. We can start from the policy formulation to enhance the continuity of the relevant expenditure policy.

### 4.4. Enhancing the Flexibility of Productive Spending Policies

Maintaining the flexibility of fiscal expenditure policy can lead to better adaptation to the dynamic changes in the complex economic situation and improve the relevance and effectiveness of government macro-control. Empirical analysis shows that productive spending has a dual impact on macroeconomic fluctuations, which can vary depending on the specific economic situation. Therefore, when applying fiscal expenditure policies, we should pay special attention to enhancing the flexibility of production-oriented fiscal expenditure policies.

The article "A Study of Fiscal Expenditure Structure and Green Economic Growth Effects: A Sample from Asian Economies" was published in 2022. Journal: J Environ Public Health.

## 5. Conclusions

Through the previous analysis, we can see that there is a strong positive correlation between the structure of fiscal expenditure and the effect of green economic growth, although on the whole, the two have a positive correlation, but for China at present, it still has a large gap compared with other developed countries. Fiscal expenditure has played an important role in the process of green economic growth in China, but there are still some shortcomings. It is clear that green finance has great potential to promote social equity and justice in the face of imperfect competition between governments and low market development, which makes it necessary for the government to make further efforts to reform and innovate in order to enhance the level of sustainability and efficiency, while also focusing on improving the efficiency of resource allocation. In order to better promote and improve the government's policy formulation and implementation of its functions, environmental protection, and resource conservation, it is inevitable that further efforts will be made to promote the optimisation and upgrading of the fiscal expenditure structure.

## Figures and Tables

**Figure 1:** Diagram of the cycle of operation of the economic and social systems.

**Figure 2:** Diagram of positive feedback mechanisms for ecological, economic, and social systems.

**Table 1:** Variable definition and descriptive statistical analysis.

Variable name	Variable definition	Mean value	Standard deviation	Crest value	Least value	Number of observations
edp	Green economy growth rate	0.108	0.095	0.415	-0.511	408
gdp	Economic growth rate	0.117	0.050	0.325	-0.047	408
Expdec	Fiscal expenditure	0.988	0.615	3.621	0.359	408
FDI	Foreign direct investment	0.026	0.022	0.146	0.001	408
k	Growth rate per capita fixed capital	0.155	0.053	0.391	-0.047	408
En	Resource endowment	4.846	3.731	25.485	0.695	408

**Table 2:** *F*-test.

	*F* null hypothesis	*F* statistics	*P* price
Fiscal expenditure for interpretation change The regression equation for quantities	*H*0 : *μi* =0	10.14	0.0001

**Table 3:** Hausman test.

	Chi-sq statistics	*F* statistics	*P* price
Fiscal expenditure for interpretation change The regression equation for quantities	10.20	0.1774	The random effects model cannot be rejected

**Table 4:** Regression results of the impact of fiscal expenditure structure on green economic growth.

Explanatory variable	edp	edp
Expdec	0.024^∗^ (1.94)	
Delivery item (FDI ∗ Expdec)	-0.032 (-0.68)	
Per capita fixed capital growth rate per capita (k)	0.229^∗∗^ (2.43)	0.292^∗∗∗^ (3.28)
Resource endowment (En)	-0.011^∗∗∗^ (-6.32)	-0.010^∗∗∗^ (-5.80)

Note: ^∗∗∗^ is a test passed at 1% significance level, ^∗∗^ is a test passed at 5% significance level, and ^∗^ is a test passed at 10% significance level.

The article "A Study of Fiscal Expenditure Structure and Green Economic Growth Effects: A Sample from Asian Economies" was published in 2022. Journal: J Environ Public Health.

**Table 5:** Comparison of regression results.

Explanatory variable	edp	edp	gdp	gdp
Fiscal expenditure	0.024^∗^ (1.94)		0.009^∗^ (1.78)	
Delivery item (FDI ∗ Expdec)	-0.032 (-0.68)		0.037^∗^ (1.87)	
Per capita fixed capital growth rate per capita (k)	0.229^∗∗^ (2.43)	0.292^∗∗∗^ (3.28)	0.392^∗∗∗^ (9.07)	0.412^∗∗∗^ (9.62)
Resource endowment (En)	-0.011^∗∗∗^ (-6.32)	-0.010^∗∗∗^ (-5.80)	-0.008^∗∗∗^ (-10.07)	-0.007^∗∗∗^ (-9.46)

Note: ^∗∗∗^ is a test passed at 1% significance level, ^∗∗^ is a test passed at 5% significance level, and ^∗^ is a test passed at 10% significance.

## Data Availability

The data used to support the findings of this study are available from the corresponding author upon request.
